The article "Discussion on the Rise of Healthy Chinese Sports Industry and the Training Mode of Compound Sports Talents" was published in 2022. Journal: J Healthc Eng.

# Discussion on the Rise of Healthy Chinese Sports Industry and the Training Mode of Compound Sports Talents

**DOI:** 10.1155/2022/6943285

**Published:** 2022-03-07

**Authors:** Hongbo Liu, Ming Li

**Affiliations:** ^1^School of Physical Education, Henan Polytechnic University, Jiao Zuo, Henan 454003, China; ^2^School of Leisure Sports, Xi'an Physical Education University, Xi'an, Shaanxi 710068, China

## Abstract

With the improvement of people's living standards and quality, sports charm stimulates people's awareness of sports consumption and makes sports industry develop rapidly into one of the important industries for the sustainable development of national economy. In modern society, sports industry has become a new industry with huge business opportunities. Especially, when the social economy develops to a certain level and sports form a certain scale, the interdependence, mutual support, and mutual promotion between sports and economy become more inseparable. This paper studies and discusses the training strategy of “compound” talents in sports industry under the background of healthy China strategy, in order to promote the development and innovation of China's sports industry. In terms of training sports talents, we should not only pay attention to personal technical, professional, practical, and understanding contents but also introduce some humanistic contents and social hot contents to improve the comprehensive quality of talents.

## 1. Introduction

With the improvement of people's living standards and quality, sports charm stimulates people's sports consumption consciousness, which makes sports industry develop rapidly and become one of the important industries for the sustainable development of national economy [1]. In modern society, sports industry has become a new industry with huge business opportunities. Especially, when the social economy develops to a certain level and sports form a certain scale, the relationship between sports and economy becomes more inseparable [2]. Sports industrialization is a part of the reform of a socialist market economy system. It is the inevitable result of the improvement of China's comprehensive national strength and the level of people's birth and death and the impact of international sports commercialization. Although China's sports industrialization started late, it has developed rapidly because it conforms to the law of economic development and meets the needs of society [3]. Only by seizing the favorable opportunity and accelerating the pace of sports industrialization can we promote the development of sports. Serving the development of national economy and promoting the construction of spiritual civilization are the key to talent training [4]. Compound talent is an important goal of talent training in China and also an important force to promote social development. In terms of sports personnel training, in addition to paying attention to personal technical, professional, practical field, and understanding-related content, we also need to introduce some humanistic content and social hot content to improve the comprehensive quality of talents [5].

The article "Discussion on the Rise of Healthy Chinese Sports Industry and the Training Mode of Compound Sports Talents" was published in 2022. Journal: J Healthc Eng.

With the improvement of China's economic development level year by year, the quality of life of residents has been greatly improved, promoting the prosperity of China's sports industry [6]. Sports industry is an industry that produces and sells sports products. It covers a wide range and has a high degree of relevance, involving many sectors of the national economy, such as construction industry, manufacturing industry, transportation and communication, food hygiene, and information services [7]. At present, the sports industry has become one of the most promising sunrise industries in the world, and with the development of the world economy and the improvement of people's living standards, the development prospect is very broad [8]. The major of physical education in colleges and universities is the cradle of cultivating sports talents. How to change the concept of physical education, strengthen the broad basic theoretical knowledge, and optimize the overall structure to broaden the professional training of physical education has been placed in front of the primary task of physical education workers [9]. Although our country has been advocating the development mode of interdisciplinary talents in the cultivation of sports talents, in the past, due to historical and social reasons, many of the cultivation modes are different from the interdisciplinary educational mode. This paper studies and discusses the training strategy of “compound” talents in sports industry under the background of healthy China strategy, in order to promote the development and innovation of China's sports industry.

Based on the healthy China strategy, this paper studies and discusses the training strategy of compound talents in sports industry so as to promote the development and innovation of China's sports industry. The main innovation of this paper lies in the cultivation of sports talents and puts forward that we can combine the school-enterprise cooperation mode to create good cooperation project opportunities, promote personal development, and maintain employment security. It will lay a foundation for the development of physical education in colleges and universities, improve the students' health level, and cultivate students' lifelong sports consciousness. By changing the concept and mode of employment, we can cultivate more innovative talents for the development of sports fitness industry and health service industry.

The article "Discussion on the Rise of Healthy Chinese Sports Industry and the Training Mode of Compound Sports Talents" was published in 2022. Journal: J Healthc Eng.

## 2. Position and Function of College Physical Education in Sports Industry

Sports and medical care are two major measures to promote human health, but their functions are different. The role of sports in health lies in how to prevent diseases, which belongs to the level of health maintenance and promotion, while the role of medical care lies in how to treat diseases, which belongs to the level of health recovery and maintenance. Due to the problems in teaching material construction and theoretical research of sports industries in China, the integration of sports and economy, sports and management, and sports and market is not enough, and the training mode of sports industry management talents has not yet been formed. The characteristics of the industry are not clear enough, and the trained talents cannot really have the ability to operate the sports industry. In the structure system of the sports industry, the sports education industry plays an important role. Physical education can create a larger output value, which is the foundation of sports industry, and it directly affects the overall development of the sports industry. The key to the benefit of sports industry is to define the products of sports industrialization and guide and standardize people's interests and behaviors with effective supervision mechanism through laws, regulations, and policies. As far as health is concerned, sports are as important as medical care. From the perspective of economic benefits, sports are even more important than medical care and should play more roles [10, 11]. Many teachers' knowledge and accomplishment in the curriculum field are worrying, and they are generally narrow minded, with a lack of knowledge and lack of understanding of the new physical education curriculum, lack of understanding of the current situation and trend of physical education curriculum reform, and lack of preparation for adapting to the new physical education curriculum reform.  Table 1, for example, shows the investigation in the field of physical education teachers' quality courses.

In many developed countries, as a pillar industry, the development of sports industry largely depends on the development of college sports industry [12, 13]. This dependence reflects the dependence of economic development in developed countries on scientific research knowledge. At the present stage of China, sports industry is a new growth point of national economy [14–16]. Therefore, the overall development of sports industry is inseparable from college physical education. The development of sports industry can not only prevent diseases and promote health but also greatly improve people's life and quality of life, especially for the elderly. A higher quality of life and physical conditions in old age will greatly improve the happiness index of people's life.

The article "Discussion on the Rise of Healthy Chinese Sports Industry and the Training Mode of Compound Sports Talents" was published in 2022. Journal: J Healthc Eng.

## 3. Current Situation and Influencing Factors of Sports Industrialization in Colleges and Universities in China

The establishment of an effective training system is the operation mechanism and management system of various training methods and human resource development technology to help enterprises achieve strategic objectives. The specific operation methods of the training mode from scratch - writing plan, setting courses, allocating resources, estimating budget and setting requirements, finally sort out and integrate, and constantly feed back and revise in practical application. In the actual operation process, some steps can be combined, which requires the trainer to use the theoretical knowledge flexibly.

As a sports culture with scale characteristics, the operation of sports industry must have its cultural and ideological basis of combining theory with practice. Compared with western developed countries, the overall development degree of college sports industry in China is still far from that of western developed countries. Professional training of compound talents is not simply to integrate professional knowledge but to comprehensively train a variety of sports-related professional knowledge. Under the cross-border requirements, it is necessary to do enough research on the contents and needs of various industries, and then integrate them into the specific training mode instead of a simple combination. At present, China lacks policies, laws, and theories supporting the industrialization of school sports, which limits the development of school sports industry. The development of sports industry in colleges and universities still lacks corresponding policies and regulations to support it. For cross-border talent training, it is important to cultivate talents' innovative ability because the innovative ability of cross-border compound talents is the ability to adapt to practical problems, which is the biggest difference between cross-border talents and ordinary talents. The development of market economy puts forward higher requirements for sports industry management, which will develop from a single administrative means in the past to comprehensive management of economic, legal, and administrative means. This requires that sports management talents not only have the ability to organize various sports activities but also have the ability to raise funds and manage sports activities, and understand the laws of market economy and sports operation.

The article "Discussion on the Rise of Healthy Chinese Sports Industry and the Training Mode of Compound Sports Talents" was published in 2022. Journal: J Healthc Eng.

## 4. Reform of “Compound” Sports Talent Training Mode in Colleges and Universities

### 4.1. Improving the Pertinence of Training Work

For the cross-border sports talent compound training mode, it should be combined with the actual training needs and the development needs of the industry to carry out targeted research. In colleges and universities, sports talents gather with complete disciplines and advanced instruments and equipment. Although in the past a long time, the scientific research ability and responsibilities of college physical education teachers have not been brought into full play, in recent years, college physical education teachers have a wider range of research topics and more diverse research methods. Under the strategy of healthy China, the applied talents needed by the health service industry must have the corresponding basic knowledge of physical education and broad knowledge of health-related disciplines. With the rise of national fitness, leisure sports, sports rehabilitation, sports tourism, and other related industries, sports talents are required to have higher sports skills, as well as certain medical and health knowledge and professional knowledge of society and management. Health promotion behavior is the end point or action result in the health promotion model, and it is a dependent variable in research. The ultimate goal of health promotion behavior is to make individuals get positive health results, enhance people's health and enable individuals and groups to achieve the purpose of health, improve and maintain health, prevent the occurrence of abnormal death, disease, and disability, improve interpersonal relationships, enhance people's self-care ability, make them get rid of superstition, abandon bad habits, develop good health habits and advocate a civilized, healthy, and scientific lifestyle, and enhance the concept of health so as to understand, support, and advocate health policies and healthy environment.  Figure 1 shows the architecture of sports talent information construction under the collaborative innovation mode.

For the training of compound talents, it is also a path and a targeted training method to carry out related comprehensive training by combining entertainment content. The reform of higher education must take the reform of educational ideology as the forerunner. Due to the poor communication, repeated allocation, and low efficiency of the competent departments of colleges and universities, the coordination among colleges and universities is not enough, and the lack of communication in the introduction of resources leads to the repeated allocation of resources. It mainly ignores the efficiency evaluation of resource input and output. And the cooperation spirit of colleges and universities is not enough. School resource management is not open enough, and the mechanism is not perfect. Colleges and universities always adhere to their own inherent operation mode in the concept of resource management. It greatly limits the competition among universities and the optimal allocation of educational resources, and it is difficult to meet the diversified needs of economic and social development. The compound model of cross-border training of sports talents has a very good promotion value for the efficiency improvement and quality assurance of the whole industry. In the process of cross border, it is necessary to provide a practical platform for talent development and provide related programs for training compound talents. With the shift of China's socialist construction center, the physical education major should be based on the height of meeting the knowledge economy era, and the training objectives and training models of this major are further studied and demonstrated in combination with the needs of today's society and quality education.

The article "Discussion on the Rise of Healthy Chinese Sports Industry and the Training Mode of Compound Sports Talents" was published in 2022. Journal: J Healthc Eng.

### 4.2. Paying Attention to the Guidance of the Cultivation Environment

For all kinds of sports colleges, we can combine the mode of school-enterprise cooperation, build good opportunities for cooperation projects, and promote personal development and good maintenance of employment security. Cross border can help talents understand the cross-border content in practice, combine entertainment, education, media, and other aspects to explore a reproducible cross-border talent training model. The content of the sports industry in colleges and universities should not be limited to physical education but should give full play to the advantages of capital and talents in colleges and universities and actively get involved in sports fitness and entertainment, sports competitions and performances, sports product management and development, and other industries. For social sports guidance and management majors and leisure sports majors, the main training goal is to train talents related to the planning and organization of sports events and the operation and management of sports industry. Therefore, outdoor sports, fitness and leisure, sports management, sports industry, sports marketing, stadium operation and management, sports event management, sports tourism, and other courses should be offered, as well as some health care courses such as fitness theory and guidance, sports injury and rehabilitation, and sports injury protection and first aid.

The article "Discussion on the Rise of Healthy Chinese Sports Industry and the Training Mode of Compound Sports Talents" was published in 2022. Journal: J Healthc Eng.

The sports industry in colleges and universities should integrate and develop together with the overall social industry, raise funds through financial allocation, self-raising by sports departments, and social fund raising, strengthen the construction of sports public welfare undertakings, and create a social atmosphere in which the whole society advocates sports and pursues a healthy lifestyle. The dimensions and overall reliability coefficient of the health-related index field evaluation system are shown in Table 2.

Applying the sports model to the input method, the system chooses a string that is most likely to be generated by solving the following decision function:

(1) $$\begin{array}{c} c_{j}\left(t\right)=\frac{1}{N}\sum_{i=1}^{N}c_{ij}. \end{array}$$

The probability of a sentence can be written as the conditional probability multiplication of 3 tuples:

(2) $$\begin{array}{c} x_{i}\left(t\right)=x\left(t\right)+n_{i}\left(t\right). \end{array}$$

Wherein the probability of each tuple is estimated by

(3) $$\begin{array}{c} x\left(t\right)=\sum_{j}c_{j}\left(t\right)+r\left(t\right). \end{array}$$

Training students' creative thinking through sports classroom teaching is conducive to promoting students' all-round development and is also an effective way to train students to feel and understand sports. The linear regression curve is calculated according to the stepwise multiple linear regression equation, as shown in Figure 2.

For cross-border development, personal ability and humanistic quality are the foundation, so it is very important to cultivate innovative ability and independent learning ability. Sports industry talents need generous knowledge, strong ability, and high quality so that they can survive and develop in the market economy. In the specific course setting process, colleges and universities should fully integrate various resources, such as increasing medical majors, sports human science, sports rehabilitation, and rehabilitation therapy, supplemented by online courses, online courses, and other teaching forms, so as to expand the scope of elective courses as much as possible and make the focus of course shift from imparting sports knowledge and skills to health promotion services.

## 5. Conclusions

Sports industrialization in colleges and universities is the inevitable outcome of further adapting to the market mechanism and the overall reform and development of colleges and universities. It will lay a foundation for the development of college sports work, improve students' health level, and cultivate students' lifelong sports awareness. Colleges and universities can combine new measures to do a good job in studying the training mode of compound talents, improve the overall training efficiency, lay a solid foundation for the development of talents and their future career, and make an important guarantee for the actual construction of China's talent echelon. The development of sports industry needs more compound sports talents to meet the professional needs. Therefore, reforming the training mode of sports talents to meet the needs of future sports industry development is an inevitable requirement for China's social and economic development and the realization of healthy China. For all kinds of sports colleges, we can combine the mode of school-enterprise cooperation, build good opportunities for cooperation projects, and promote personal development and good maintenance of employment security. Under the strategy of healthy China, the applied talents needed by the health service industry must have the corresponding basic knowledge of physical education and broad knowledge of health-related disciplines. Talent training of physical education majors in colleges and universities should not only pay attention to students' employability but also pay attention to students' innovative and entrepreneurial abilities. By changing employment concepts and employment methods, more innovative talents can be trained for the development of sports fitness industry and health service industry.

The article "Discussion on the Rise of Healthy Chinese Sports Industry and the Training Mode of Compound Sports Talents" was published in 2022. Journal: J Healthc Eng.

## Figures and Tables

**Figure 1:** System structure of sports talent information construction.

**Figure 2:** The relationship between the actual value and the calculated value of stepwise linear regression.

**Table 1:** The survey of physical education teachers' quality courses.

	Curriculum view	Curriculum resources	Curriculum implementation	Curriculum evaluation	Curriculum reform
Average score	8	7	11	9	6
Accuracy (%)	50.8	45.5	68.6	57.7	55.3

**Table 2:** Various dimensions and overall reliability coefficients of the health-related finger field evaluation system.

Dimensions	Number of indicators
Activity ability	17
Somatic function	7
Emotional character	11
Memory function	4
Healthy behavior	8
Social adaptability	5

## Data Availability

The data used to support the findings of this study are included within the article.
